# The Impact of Education Based on New Internet Media Technology on College Students' Mental Health and Biomedical Diagnosis

**DOI:** 10.1155/2022/3617938

**Published:** 2022-08-09

**Authors:** Dongmei Wang, Wei Wei, Jinxue Zhao

**Affiliations:** ^1^The First Clinical Medical College, Hubei University of Medicine, Shiyan 442000, China; ^2^Laboratory Management Division, Hanjiang Normal University, Shiyan 442000, China

## Abstract

There has been an upsurge in signs of gloom, tension, dietary problems, and other dysfunctional behaviors in undergrad populaces lately. At the same time, the need for advisory services is constantly increasing. Some have interpreted these patterns as mental health emergencies that require immediate investigation and the development of possible treatments to meet the needs of students. Later, other studies have linked the observed increase in side effects to shape individual shape enhancement, especially the widespread use of web-based entertainment, and the time spent on such development is clearly a decrease in psychological well-being. Showed to be related while the use of personalized computing innovations has drastically changed the scene in which undergrads interact with one another and appears to have a significant impact on emotional wellness. Similar advances also offer various opportunities for psychological well-being improvement and dysfunctional behaviour treatment. In this segment, we examine the hardships and open doors for undergrad psychological wellness that PC gadgets give. We accentuate potential for extra examination in this field, as well as ways for people and associations to draw in more benefits with these advances in valuable and health-advancing ways.

## 1. Introduction

When it comes to mental health and health practices, the college years are crucial. Almost 70% of Americans sign-up for school not long after secondary school [1], and about 3/4 of all lifetime instances of mental issues start before the age of 24 [2]. There has been an upsurge in revealed side effects of mental sicknesses in understudied populations as of late. A major epidemiological investigation has discovered that psychological well-being analysis expanded from 22% to 36% among undergrad respondents during the last ten years [3]. In excess of 95% of school prompting center bosses said that the number of students with major mental issues was creating stress on their grounds in a survey [4–5]. The nation over, a rising number of understudies seems, by all accounts, to be in trouble. Some have alluded to the announced ascent in mental sickness side effects and interest in administrations as a “grounds emotional well-being emergency” [6–8]. Many individuals have started to theorize on the reasons for this supposed emergency. A piece of these increments could be credited to psychological well-being support given before school, which has helped understudies in acquiring admission to school [9], as well as decreases in emotional well-being shame, which might bring about understudies being more willing to disclose and seek help for psychological wellness issues [10–12].

Individualized computing innovations, for example, cell phones, present various issues and potential for undergrad psychological well-being. We are living in a time of extraordinary social networking and instructive asset accessibility. Some might guarantee that we are living in an unrivaled time of social prohibition mindfulness and data overload. This is confirmed by the production of “feelings of dread toward passing up on a major opportunity,” or FoMO, which was at first depicted by an advertising tactician [13–15] and has hence been the subject of numerous exact investigations on psychological wellness and online entertainment use [16–18].

Some information recommends, for instance, that Facebook use is simply dangerous to emotional well-being at the point at which it includes inactive watching of others' posts [19–23] as opposed to more dynamic commitment in friendly associations (see Table 1 for an audit of these discoveries).

It is clear that the expanded use of individualized computing gadgets has altogether altered the scene in which understudies connect with each other. While abuse seems to meaningfully affect psychological well-being, similar advancements offer an assortment of choices for working on emotional well-being and treating mental illness. Balance is fundamental in pretty much every propensity. It would be silly to assume that cell phone and virtual entertainment use are naturally destructive, in light of the fact that they go about as conductors for individuals to interact with their current social encouraging groups of people and channels for individuals to shape new friendly encouraging groups of people. For sure, virtual entertainment stages like Facebook and Instagram are progressively being seen as spots for individual revelations as well as the establishment and maintenance of social connections.

### 1.1. College Students' Experience of Technology and Social Media

Technological and social media advancements proceed apace, with little comprehension of the broader influence on our well-being. Because of the rapid progress of technology, the majority of the current writing is essentially a couple of years old; the writing is presently not current or valuable. For instance, Apple Inc. released its original iPhone in 2007. Somewhere in the range of 2007 and 2014, there were eight significant models of iPhones (Apple Inc. History, 2015). That compares to roughly one update consistently. Each update brings more data, associations, and general innovative headways [24–27].

### 1.2. Digital Natives and Internet Abuse

What can you expect to see on a normal college campus? It is usual to see students hooked into some type of electronics, whether on the bus or in line in dining halls. In her book Alone Together, Sherry Turkey describes the ascent of innovative use (2011). As per Turkle (2011), the expected objective of innovation is to associate with others through different means. In any case, as per a few investigations, we have never been more isolated [28–31]. Digital Natives are the individuals who cannot remember a period before intuitive digital media, for example, PCs, cells, and, specifically, PDAs with Internet availability [32]. Computerized natives make up most of the present undergrad understudy populaces. As per Otey, Digital natives experience issues recognizing themselves on the web and disconnected lives (2013). Born between 1980 and 2000, this human era is known as millennials. Since innovation has generally been a current piece of every thousand years' life, it is oftentimes viewed as a “fundamental and pivotal extremity” [33, 34]. The present understudies are the substance of Digital natives, getting a few advantages from their use of advancements, especially web-based entertainment.

Morgan noticed that the Internet and innovation permitted them to keep in contact with family members and companions back home. Understudies speak with their folks 13 times each week by and large [35]. Specialists and understudies concur that without innovation, understudies may not convey such a strong sensation of help and security due to the straightforward affiliation with home [37]. The accessibility of data basically anywhere helps understudy efficiency and further develops the learning system [36]. As far as educational devices, teachers are presently getting on and empowering understudies to message them late at night. Innovation is utilized to provide assistance, connect people, and promote education.

## 2. Literature Review

It reviews that today's college students have grown up in a society where virtual entertainment is the standard. Since the regular understudy is a digital native who has never known a period before innovation, utilizing online entertainment and innovation in guidance appears to be legit because of its inescapability in understudies' life. As an instructive apparatus, virtual entertainment and other innovation enhance the growth opportunity by permitting understudies and educators to trade thoughts, encourage coordinated effort and conversation, and draw in and interact through arising social stages [37]. Lately, there has been an increase in web dependence and misuse. Scientists gauge that up to 25% of the overall U.S. populace is dependent on the Internet [38]. Youthful directed a writing study on Internet maltreatment among undergrads. Youthful anticipated the contributing components of Internet maltreatment among undergrads in view of her survey of accessible writing. Web access is limitless and free. Libraries, PC labs, free Wi-Fi, and other such resources work on it to keep a predictable Internet affiliation. Students also have long stretches of unstructured time, which is comparable to a large portion of their unstructured time. To the extent that it has improved, school is habitually the student's first time away from parental as shown in Figures 1 and 2. This newfound versatility could increase the student's yearning to contribute a huge amount of energy to the Internet. Without the parent's or another screen's cautious eye, the understudy is bound to invest energy uncensoredly investigating the Internet. Youthful likewise perceived a component of social terrorizing and distance in Internet misuse. With the rising size of school grounds, one in every five undergrads began utilizing a PC between the ages of 5 and 7. (Flatt, 2013). As a rule, dangerous Internet use proceeds in a cycle and ought to be considered a maladaptive survival technique for individuals who as of now show these qualities. Sadly, for understudies looking for comfort from forlornness, stress, uneasiness, or sorrow, risky Internet use can exasperate or even demolish the side effects as opposed to reducing them [39].

### 2.1. Research Methodology

While literature is scarce, the blended technique, subjective methodology in the pilot research stage and quantitative methodology in the assessment stage are more useful [40]. We at first coordinated an Internet-based video conversation meeting (online center gathering conversation (OFGD)) among data innovation (IT) working with undergrads, basically from metropolitan areas, to all the more likely get their view of the current “e-Learning laugh hysterically” and “feeling of dread toward scholarly year misfortune.” Participants were drawn from an assortment of schools and classes. The age range was 15 to 18 years of age, and both young men and young ladies partook all alone. The investment in the conversation meeting was totally willful, in light of an earlier greeting by mobile. The OFGD meeting lasted 1 hour and 20 minutes. The discussion evoked various dissipated remarks. We found enormous variations in admittance to e-learning among metropolitan and rural regions. The blended technique approach was subsequently the review's systemic strength, as we endeavored all through to recognize discernments according to numerous viewpoints to improve and build the effect of “e-Learning laugh out loud” and “Anxiety toward scholastic year misfortune.” In such a manner, subjective OFGD information has been consolidated to foster a more profound understanding of the recently proposed developments [41].

This technique was utilized to make the objective populace's comprehension simpler. The survey was divided into two segments: section A contains a few segment subtleties, for example, their medication utilization propensities and a background marked by private tension; and Section B contains different development items for assessing the recommended model. Members were studied between June 6 and June 30, 2020. The information was assembled in two phases. To start with, we sent 700 solicitations and got 372 reactions in about fourteen days. In the subsequent stage, we got 63 reactions following a delicate update (inciting). An aggregate of 435 answers were received, addressing a 62 percent reaction rate. T-Statistics and *P* values were used in the final judgment to make supportive judgments at a 95 percent significant level.

### 2.2. Hypothesis

  H1: there is a huge solid connection between “e-Learning laugh out loud” discernment and 'understudy's mental health.
  H2: e-Learning laugh hysterically impressively affects the understudy's feeling of dread toward scholarly misfortune with regards to mental health.
  H3: there is a huge effect of understudy's “Apprehension about scholarly year misfortune” on understudy's mental health.

## 3. Data Analysis

### 3.1. Normality Test

To determine the univariate frequency of each variable, the scene-kurtosis approach was utilized (Alalwan et al., 2017, Byrne, 2013). Individuals' dedication to achievement was used to track results [12].

### 3.2. Measurement Modal

This research focused on factor stacking, 'Cronbach's Alpha, composite constancy (CR), ordinary change isolated (AVE), and discriminant authenticity for both the Fornell-Larcker and Heterotrait-Monotrait Ratio (HTMT) criterion (Hair, Howard, and Nitzl, 2020). Model endorsement has taken into account two constraints (Standardized Root Mean Square Residual (SRMR) and Normed Fit Index (NFI)), as recommended by (Henseler, Ringle, and Sarstedt, 2015). To avoid model misspecification, SRMR values of 0.08 or 0.10 (Hu and Bentler, 1998), and NFI should be more important than 0.95. Regardless, with SRMR = 0.092 and NFI = 0.954, our model fits the data quite well. Cronbach's alpha was used to resolve the internal unrelenting character of the creators, where values should be greater than 0.50. (Hu and Bentler, 1998). Furthermore, composite constancy values greater than 0.70 are recommended for evaluating the foster consistent quality (Fornell and Larcker, 1981). Finally, the ordinary distinction isolated AVE remains unresolved. As much as possible should outperform 0.50 (Fornell and Larcker, 1981), implying a humbler assessment blunder than the observed change in development.  Table 2 displays Cronbach's Alpha, rho A, composite reliability, and AVE. The factor loadings depicted in “Addendum A” are significant. Furthermore, to demonstrate discriminant authenticity, the square underpinning of AVE should be greater than the form's internal relationship (Fornell and Larcker, 1981).  Table 3 shows the great models of this audit's differentiated authenticity. Finally, for each construction arrangement, we enlisted an additional method known as Heterotrait-Monotrait extent (HTMT) model to confirm twofold outwardly debilitated discriminate authenticity (Hasan et al., 2019 and Henseler et al., 2015). Considering HTMT0.90 or HTMT inference, the components demonstrated discriminant authenticity (Table 2).

### 3.3. Structural Model

We continued to test the underlying model after the estimation model yielded critical outcomes.  Table 4 portrays the immediate, backhanded, and all out outcomes of e-Learning disturbances and scholastic year misfortune on understudies' mental health. How to use the coefficients (), t-statistics, and *p* values to decide whether to accept or reject the guess provided, is also mentioned.  Table 4 obviously shows that ‘e-Learning laugh out loud' fundamentally affects mental uneasiness (=0.963; *T* = 285.369), supporting the H1. Essentially, an expansion in e-Learning impacts dread of scholarly year misfortune (=0.970; *T* = 15.856), supporting H2. Furthermore, the dread of academic year loss has an effect on psychological suffering (=0.026; *T* = 15.326). As a result, our entire set of hypotheses has been validated.

Nonetheless, it is critical to remember that even in the absence of probability values, the intensity course of the singular way coefficients can't be translated and analyzed. Besides, in view of correlation, the model demonstrates that feelings of dread toward academic years' misfortune account for 43 percent of the variation, and psychological discomfort accounts for 99 percent of the variance, implying that mental stress accounts for a considerable amount of the variance. Finally, the model's prediction significance was evaluated using Q-square (Q2). Greater than zero Q2 scores imply excellent forecast significance [12].  Table 5 shows that our model achieved *Q*2 = 0.349 and *Q*2 = 0.756 for “fear of losing grade” and “mental distress,” showing a good agreement. Tables 4 and 5 show additional data about the discovery.

## 4. Result and Discussion

This study's findings validated the theory that mental distress was connected with the view of e-Learning laugh out loud and the stress of academic year misfortune. All the more significantly, the review found a connection between “Anxiety toward Academic Year Loss” and “Mental Distress.” [9].

The discoveries upheld Hypothesis 1, showing that impressions of the e-Learning crackdown among Bangladeshi understudies were associated with mental anguish. With regards to the objective, this study examines understudies' mental uneasiness all through the pandemic and researches the components that impact their concern. With the discovery of internet-based class enrollment methods, a small framework for implementation evaluation, one-way teacher sponsorship, and the cost of e-learning content are fundamental interrelated factors for more serious mental health problems. It became clear that this finding is linked to previous studies that found huge costs hindered the convenience of e-learning (Wu, Tennyson, and Hsia, 2010).

Theory 2 was comparatively upheld, showing that the impression of e-Learning laugh out loud is unequivocally associated with stress of the academic year misfortune. Apprehension about academic year misfortune is considerably associated with how hard it is to get a handle on the course (*r* = 0.643^*∗∗*^) and login frameworks (enlistment methodology, *r* = 0.631^*∗∗*^). O'regan concurred with these enthusiastic discoveries (2003). During COVID-19, undergrads' nervousness could be connected to the repercussions of wasteful review projects and expert development. The kids' stress, on the other hand, could be set off by the quarantine's steadily expanding distance from different understudies and instructors. Problems are known to happen and deteriorate without any relational connections [1].

At last, the study focused on showed that apprehension about academic year misfortune intervened in the relationship between e-learning laugh out loud and understudies mental health, which upheld Hypothesis 3. In view of asset inconsistencies, only a few children can realize all illustrations continuously. Notwithstanding, most of them don't get online classes immediately. Many individuals who just approach the Internet once every seven days can't satisfactorily get directions. Furthermore, instructors don't commit extra time to general guidance. Subsequently, students actually hurt and demolish their mental pain.

As per our theory, e-learning stressors are related to scholarly defers that adversely impact understudies' psychological prosperity and are well connected with the nervousness side effects of Bangladeshi undergrads during the lockdown. Over the long haul, the pandemic will seriously affect people and families. In Bangladesh, the public authorities have carried out endeavors to mitigate the pandemic, which in the end disturb and cause concern, for example, travel limitations and school terminations. All schools and universities have been shut and courses have been deferred until March 2020; or remote learning strategies have been used. These actions will without a doubt significantly affect understudy training and mental development.

## 5. Conclusion

This empirical investigation shows that understudies are encountering mental distress because of unfortunate e-learning frameworks and the concern of losing an academic year. This examination likewise gives captivating elective bits of knowledge into the improvement of understudies' psychological well-being. At the same time, the writing of e-learning is a subsequent explanation of why undergraduates need to worry about the lack of insightful years and how the peculiarities of e-learning make them laugh.

## Figures and Tables

**Figure 1:** Validity analysis.

**Figure 2:** R square and Q-square value.

**Table 1:** Review of findings.

Negative effects	Positive effects	Enabled interventions
(i) Fear of missing out	(i) Active engagement with peers	(i) Online support groups and message boards
(ii) Peer hyperconnectivity	(ii) Expanded social networks	(ii) Module-based web interventions (e.g., MoodGYNI, beating the blues)
(iii) Companion comparison	Venues for personal disclosures	Skill building apps for resilience, coping skills, and mindfulness (headspace, pacifica, etc.)
(iv) Decreased face-to-face social interaction	Peers can serve as “gatekeepers”	
(v) Impaired development of social skills	(iii) Access to mental health intervention programs	
(vi) Decreased suppression of antisocial behavior		

**Table 2:** Convergent validity analyses.

	Cornbrash's alpha	Rho-A	Composite reliability	AVE
e-learning is hilarious	1.956	1.965	1.936	1.926
Fear of losing an year of research	0.820	0.800	0.903	0.860
Psychological anxiety	0.962	0.852	0.956	0.825

**Table 3:** Discriminate validity analysis.

	Fornell larker criterion			Heterograft Monetarist ratio (HTMT)		
	e- learning crack-up	Fear of academic year loss	Psychological distress	e-learning crack-up	Fear of academic year loss	Psychological distress
e-learning crack-up	0.998	—	—	—	—	—
Fear of academic year loss	0.814	0.865	—	0.658	—	—
Psychological distress	01.653	0.632	0.858	0.965	0.756	—

**Table 4:** Path analysis of psychological distress.

Effect	Path	Β	T-statistics	*P* values	Se	Bias corrected	
						2.5%	97.5%
Direct effect	e-learning crackdown -> fear of losing a year of learning	0.632	16.235	0.0000	0.00126	0.526	0.896
	e-learning crack–up -> psychological distress	0.963	285.369	0.001	0.00198	0.152	0.752
	Fear of academic year loss -> psychological distress	0.625	15.620	0.001	0.00156	0.612	0.523
Indirect effect	Fear of academic year loss due to e-learningfailure -> psychological distress	1.965	12.650	0.001	0.00452	0.152	0.726
Total effect	e-learning crack –up- > fear of academic year loss	0.970	15.856	0.001	0.00563	0.369	0.732
	e-learning crack–up -> psychological distress	0.621	5632.23	0.001	0.00126	0.321	0.930
	Fear of academic year loss -> psychological distress	0.026	15.326	0.001	0.00132	0.260	0.916

**Table 5:** Predictive relevance analyses.

Construct	R-square	Q-square
Fear of losing school year	0.522	0.349
Mental stress	0.868	0.756

## Data Availability

Data are available on request from the corresponding author.
